RETRACTED

# MicroRNA‐769‐5p suppresses cell growth and migration via targeting NUSAP1 in bladder cancer

**DOI:** 10.1002/jcla.23193

**Published:** 2020-01-03

**Authors:** Yifan Chen, Wentao Zhang, Aimaitiaji Kadier, Haimin Zhang, Xudong Yao

**Affiliations:** ^1^ Department of Urology Shanghai Tenth People's Hospital Tongji University Shanghai China

**Keywords:** cell growth, invasion, migration, miR‐769‐5p, nucleolar and spindle‐associated protein 1

## Abstract

**Background:**

Nucleolar and spindle‐associated protein 1 (NUSAP1) has been identified to be strongly implicated in the carcinogenesis of cervical carcinoma, breast cancer, and liver cancer, and shows a high expression level in bladder cancer, indicating that NUSAP1 might be a potent target for cancer treatment. Using bioinformatics methods, we found that NUSAP1 was a putative target of miR‐769‐5p. Here, we aimed to explore whether miR‐769‐5p is involved in bladder cancer progression via targeting NUSAP1.

**Methods:**

MiR‐769‐5p expression patterns in bladder cancer tissues and cells were detected by RT‐PCR. Kaplan‐Meier was used to determine the clinical effects of miR‐769‐5p expression levels on the overall survival of bladder cancer patients. Bioinformatics methods were used to predict the binding sites between miR‐769‐5p and NUSAP1, which was verified by the luciferase gene reporter assay. CCK‐8, flow cytometry, wound healing and transwell chamber experiments were performed to test cell growth, apoptosis, migration and invasion capacities.

**Results:**

miR‐769‐5p was lowly expressed in bladder cancer tissues and cells, which was closely associated with poor prognosis. Overexpression of miR‐769‐5p induced significant repressions in cell growth, migration, and invasion and caused an obvious increase in cell apoptosis, whereas these tendencies were reversed when NUSAP1 was upregulated.

**Conclusion:**

This study demonstrates that miR‐769‐5p functions as a tumor suppressor in bladder cancer via targeting NUSAP1.

## 1 INTRODUCTION

Bladder cancer is the most common malignant tumor occurring in the urinary system and accounts for one of the most prevalent malignancies all over the world.^1^ Based on the depth of tumor invasion, bladder cancer can be divided into non–muscle‐invasive tumor and muscle‐invasive tumor which accounts for about 20%‐30%.^2^ Approximately 30% of patients with of muscle‐invasive tumor are associated with distant metastasis at the time of diagnosis, with an unsatisfactory 5‐year survival rate.^3^ Therefore, it is a necessary need to find novel biomarkers and therapeutic targets for bladder cancer.

Nucleolar and spindle‐associated protein 1 (NUSAP1) is a microtubule‐binding protein and has been found to play important roles in mitotic spindle assembly.^4^ The expression of NUSAP1 is frequently increased in the proliferating cells, leading to microtubule bundling and G2/M phase arrest.^5^ Recently, reposts have demonstrated that NUSAP1 is strongly implicated in the tumorigenicity of several kinds of cancers, such as cervical carcinoma,^6^ breast cancer,^7^ and liver cancer.^8^ In bladder cancer, Pan et al^9^ reported that NUSAP1 was overexpressed in bladder cancer and play crucial roles in the maintain of stemness in bladder cancer cells. However, the detailed mechanisms underlying NUSAP1 in bladder cancer progression still remain unknown.

RETRACTED

MicroRNAs (miRNA) are a class of small non‐coding RNAs with about 20 nucleotides. It is well documented that miRNAs can induce translation degradation or repression, thereby cause mRNA silence via bind to the complementary recognition sequences in their targeted mRNAs.^10^ Via targeting target mRNAs, miRNAs exert important roles in carcinogenesis via regulating multiple biological functions, including cancer cycle, proliferation, survival, invasion, angiogenesis, and epithelial‐mesenchymal transition (EMT).^11^, ^12^, ^13^ Bioinformatics method predicts that NUSAP1 is a target of miR‐769‐5p, but whether miR‐769‐5p is involved in bladder cancer progression via targeting NUSAP1 need to be elucidated.

In this study, we aimed to explore the functions of miR‐769‐5p/NUSAP1 axis in the progression of bladder cancer in vitro.

## 2 MATERIALS AND METHODS

### 2.1 Bladder tissue samples

Ninety‐six bladder cancer tissues and the paired peritumoral normal bladder tissues were derived from patients with bladder cancer who received bladdertomy in Shanghai tenth people's hospital between February, 2015 and February, 2018. The informed consent has been obtained from every patient. This study has been performed in accordance with the Helsinki Declaration and was approved by the ethical committee of Shanghai tenth people's hospital.

### 2.2 Cell lines and culture conditions

The epithelial immortalized uroepithelium cell line SV‐HUC‐1 and 3 bladder cancer cell lines, such as HT‐1376, 5637 and T24 were purchased from American Type Collection Culture (ATCC). SV‐HUC‐1 cells were grown in F‐12K Medium (ATCC); HT‐1376 cells were cultured in Eagle's Minimum Essential Medium (EMEM, ATCC); 5637 cells were grown in RPMI‐1640 medium (ATCC) and T24 cells were cultured in McCoy's 5a medium (ATCC), supplemented with 10% fetal bovine serum (FBS; Gibco).

### 2.3 Cell transfection

The mimic and inhibitor used to overexpress and silence miR‐769‐5p in bladder cancer cells, together with the negative control vectors (mimic‐NC, inhibitor‐NC) were synthesized by GenePharma. The plasmid applied to upregulate NUSAP1, called as OE‐NUSAP1 and OE‐NC were purchased from OriGene (No. SC327860). For cell transfection, HT‐1376 and T24 cells were inoculated in 6‐well plates and cultured at 37°C overnight, followed by cell transfection with the above vectors using Lipofectamine 2000 (Invitrogen) referring to the manufactory's descriptions.

RETRACTED

### 2.4 Quantitative real‐time PCR (RT‐PCR) analysis

Total RNA extracted from cells using the RNApure Tissue & Cell Kit (DNase I) in accordance to the manufacturer's instructions (CWBIO). Then, a total of 1 μg RNA were submitted to the reverse transcription of miRNA and mRNA using stem‐loop primers and random primers with TaKaRa system according to the manufactory's instructions. Subsequently, the RT‐PCR was carried out using a TaqMan Universal Master Mix II kit on a Bio‐Rad detection system (Bio‐Rad). GAPDH and U6 expression levels are served as internal references to normalize mRNA and miRNA expressions, respectively. Primers were listed as follows.

NUSAP1: forward (F)‐5′‐ ACCAGACGAGCACCAAGAAG‐3′; Reverse (R)‐5′‐ ATTGATGGGCTGCTGCTTCA‐3′; GAPDH: F‐5′‐ CCACTAGGCGCTCACTGTTCTC‐3′; R‐5′‐ ACTCCGACCTTCACCTTCCC‐3′

### 2.5 Western blotting assay

Total protein extraction was carried out by using the RIPA lysis buffer (Sangon Biotech, Shanghai, China) with protease inhibitor (Solarbio), according to the manufactory's description. After quantification with a BCA Protein Kit (Bio‐Rad Laboratories), 30 μg proteins of each sample were separated by 10% polyacrylamide gels and were transferred to polyvinylidene difluoride membranes (Millipore). The membranes were then incubated with 5% non‐fat milk and probed with the primary antibodies overnight at 4°C, including NUSAP1 (1:1000 dilution; No. ab137230, Cambridge, MA, USA), Bcl2 (1:1000 dilution; No. #15071, Cell Signaling Technology), Bax (1:1000 dilution; No. #2772, Cell Signaling Technology), E‐cadherin (1:1000 dilution; No. #3195, Cell Signaling Technology), N‐cadherin (1:1000 dilution; No. #4061, Cell Signaling Technology), and GAPDH (1:2000 dilution; No. #2118, Cell Signaling Technology). After the incubation with the corresponding second antibodies (Santa Cruz Biotechnology), the protein expression levels were determined on a Western blotting imaging and quantitative system (Bio‐Rad). Protein quantification was performed using the ImageJ software (National Institutes of Health) after background subtraction, with GAPDH level as an internal reference.

### 2.6 Luciferase gene reporter assay

The putative binding sites between miR‐769‐5p and NUSAP1 were predicted using TargetScan (http://www.targetscan.org/vert_71/) and miRDB (http://www.mirdb.org/index.html). The wild‐type and the mutant type of the 3’UTR NUSAP1 were cloned into pGL3 vector (Promega), which were called as WT or MUT, respectively. For luciferase gene reporter assay, HT‐1376 and T24 cells were co‐transfected with WT/MUT and mimic‐miR‐769‐5p/mimic‐NC. The luciferase activity was determined through a dual‐luciferase assay system (Promega) in referring to the manufacturer's descriptions.

RETRACTED

### 2.7 Cell Counting Kit‐8 assay (CCK‐8)

CCK‐8 assay was used to detect cell proliferation. In brief, HT‐1376 and T24 cells were seeded in 96‐well plates at a density of 3 × 10^3^ cells/well and cultured at 37°C overnight, then the cells were given different cell transfections. After incubation at 37°C for the indicated times, culture medium was replaced with 10 μL CCK‐8 reagent (Beyotime) and 90 μL fresh medium, and incubated at 37°C for another 4 hours. The absorbance at 450 nm was measured with a plate reader (model 680; Bio‐Rad).

### 2.8 Flow cytometry assay

Flow cytometry assay was carried out to detect cell apoptosis. In brief, HT‐1376 and T24 cells transfected with different vectors were harvested and subjected to apoptosis detection using Annexin V(FITC)/Propidium iodide (PI) Apoptosis Detection Kits (Dojindo). Cell apoptosis rate was detected by using flow cytometry (Beckman Coulter) and analyzed using FlowJo 7.6 software (Tree Star, lnc).

### 2.9 Wound healing assay

Wound healing assay was used to assess cell migration ability. In brief, HT‐1376 and T24 cells were plated in 6‐well plates at a concentration of 5 × 10^5^ cells/mL and cultured at 37°C overnight, followed by different cell transfections. The wounds were made using 20 μL pipette tips when cell confluence being reached at 100%, and the gloating cells were removed via PBS washing. Then, the cells were cultured at 37°C with 60% H_2_ administration or not. Images of cells movement to the scratch area were taken every 6‐12 hours using a microscope.

### 2.10 Transwell chamber assay

Transwell chambers with 8‐μm polycarbonate filters (BD Bioscience) were applied for cell invasion assessment. In procedure, chambers were coated with Matrigel on the lower side. Then, approximately 2 × 10^5^ HT‐1376 and T24 cells resuspended with FBS‐free medium were seeded in the upper chamber, while 600 μL medium supplemented with 20% FBS was added into the lower chamber. Following 48 hours of incubation at 37°C with 5% CO_2_ or 60% H_2_, cells in the top of the membranes were removed using cotton buds and cells at the bottom of the membrane were fixed and stained with 0.2% crystal violet (Solarbio). The stained cells were counted under a light microscope (magnification: 200×) to assess cell invasiveness.

RETRACTED

### 2.11 Statistical analysis

Each experiment in the current study was performed in triplicate. Statistical significance comparison between two groups and multiple groups was carried out using student's *t* test and one‐way ANOVA, respectively. Data analysis was performed by using GraphPad Prism (version 6.0). *P* < .05 was considered as statistical significance.

## 3 RESULTS

### 3.1 miR‐769‐5p is lowly expressed in bladder cancer tissues and cells and closely associates with the poor prognosis

To reveal the functions of miR‐769‐5p/NUSAP1 axis in the progression of bladder cancer, we first explore the expression patterns of miR‐769‐5p in bladder cancer tissue samples. miR‐769‐5p showed a low expression pattern in the cancer tissues as compared with the paracancerous tissues, as detected by the RT‐PCR assay in 96 paired cancer tissues and normal tissues (Figure 1A). miR‐769‐5p low expression predicted shorter overall survival in patients with bladder cancer (Figure 1B‐C). In addition, miR‐769‐5p expression was significantly decreased in bladder HT‐1376, 5637, and T24 cell lines when compared to that in the normal bladder SV‐HUC‐1 cell line (Figure 1D). These findings suggest that miR‐769‐5p might play a role in the progression of bladder cancer.

**Figure 1:** Evaluation of the expression pattern and clinical value of miR‐769‐5p in bladder cancer. A, RT‐PCR analysis of the expression levels of miR‐769‐5p in 96 paired bladder cancer tissues and normal tissues. B, Kaplan‐Meier analysis of the relationship between miR‐769‐5p expression levels of the overall survival in bladder cancer. C, TCGA predicted the clinical value of miR‐769‐5p expression patterns in bladder cancer prognosis. D, RT‐PCR analysis of the expression levels of miR‐769‐5p in SV‐HUC‐1, T24, HT‐1376, and 5637 cells. (^*^ *P* < .05)

### 3.2 miR‐769‐5p functions as a tumor suppressor in bladder cancer

Next, we carried out the gain/loss‐of‐function assays to investigate miR‐769‐5p roles in the progression of bladder cancer in vitro. Transfection with mimic‐miR‐769‐5p significantly increased miR‐769‐5p expression while inhibitor‐miR‐769‐5p transfection decreased miR‐769‐5p expression in both T24 (Figure 2A) and HT‐1376 (Figure 2D) cell lines. Upregulation of miR‐769‐5p caused significant repressions in cell growth (Figure 2B,E), invasion (Figure 2G,I), and migration (Figure 2H,J) while an increase in cell apoptosis population (Figure 2C,F) in both T24 and HT‐1376 cell lines, indicating that miR‐769‐5p serves as a tumor suppressor in bladder cancer.

**Figure 2:** Assessment of miR‐769‐5p roles in bladder cancer progression. T24 and HT‐1376 cells were transfected with mimic‐NC, mimic‐miR‐769‐5p, inhibitor‐NC, or inhibitor‐miR‐769‐5p and were subjected to the following assays. A, RT‐PCR analysis of the expression of miR‐769‐5p in T24 cells. B, CCK‐8 analysis of cell growth in T24 cells. C, Flow cytometry assay was used to assess cell apoptosis in T24 cells. D, RT‐PCR analysis of the expression of miR‐769‐5p in HT‐1376 cells. E, CCK‐8 analysis of HT‐1376 cell growth. F, Flow cytometry assay was used to assess HT‐1376 cell apoptosis. G, Transwell chambers were applied to assess T24 cell invasion. H, Wound healing assay was used to assess T24 cell migration. I, Transwell chambers were applied to assess HT‐1376 cell invasion. J, Wound healing assay was used to assess HT‐1376 cell migration. (n = 3, ^*^ *P* < .05, compared with mimic‐BC group; ^#^ *P* < .05, compared with inhibitor‐NC group)

RETRACTED

### 3.3 NUSAP1 is a target of miR‐769‐5p and is upregulated in bladder cancer

Using bioinformatics method, we found that NUSAP1 was a direct target of miR‐769‐5p and Figure 3A showed the putative binding sites. Overexpression of miR‐769‐5p significantly decreased the luciferase activity of WT, whereas this effect was abolished when the binding sites were mutated (Figure 3B‐C). In addition, the bioinformatics software starBase showed that NUSAP1 was highly expressed in bladder cancer (Figure 3D), which was closely associated with the poor prognosis in bladder cancer (Figure 3E). Moreover, RT‐PCR and Western blotting confirmed the inhibitory effect of miR‐769‐5p on NUSAP1 expression, which was reversed when NUSAP1 was overexpressed (Figure 3F‐I). Overall, these findings indicate that NUSAP1 is a direct target of miR‐769‐5p in bladder cancer.

**Figure 3:** Evaluation of the relationship between miR‐769‐5p and NUSAP1. A, The putative binding sites between miR‐769‐5p and the 3'UTR of NUSAP1 mRNA. B‐C, Luciferase gene reporter assay was used to evaluate the luciferase activity of MUT/MT after cells were transfected with mimic‐NC/mimic‐miR‐769‐5p (n = 3, ^*^ *P* < .05). D, StarBase predicted NUSAP1 expression patterns in bladder cancer tissues and normal tissues. E, StarBase predicted the clinical value of NUSAP1 expression patterns in bladder cancer prognosis. F‐G, RT‐PCR analysis of the mRNA levels of NUSAP1 in T24 and HT‐1376 cells transfected with mimic‐NC + OE‐NC, mimic‐miR‐769‐5p + OE‐NC, mimic‐miR‐769‐5p + OE‐NUSAP1 or mimic‐NC + OE‐NUSAP1. H‐I, Western blotting analysis of the protein expression level of NUSAP1 in T24 and HT‐1376 cells transfected with mimic‐NC + OE‐NC, mimic‐miR‐769‐5p + OE‐NC, mimic‐miR‐769‐5p + OE‐NUSAP1, or mimic‐NC + OE‐NUSAP1 (n = 3, ^*^ *P* < .05, compared with mimic‐NC + OE‐NC group; ^#^ *P* < .05, compared with mimic‐miR‐769‐5p + OE‐NC group)

RETRACTED

### 3.4 miR‐769‐5p represses bladder cancer progression via targeting NUSAP1

We then explored the effects of miR‐769‐5p/NUSAP1 axis on the progression of bladder cancer in vitro. The results showed that NUSAP1 overexpression apparently rescued miR‐769‐5p‐mediated inhibitions in cell growth (Figure 4A,D), invasion (Figure 4C‐F), and migration (Figure 4G‐H), as well as the promotion in cell apoptosis (Figure 4B,E). Furthermore, overexpression of miR‐769‐5p significantly decreased the expression of Bcl2 and N‐cadherin and increased Bax and E‐cadherin expression, whereas this effect was abolished when NUSAP1 expression was upregulated in both T24 and HT‐1376 cell lines (Figure 5A‐B). The above results confirm that miR‐769‐5p functions as tumor suppressor in bladder cancer via targeting NUSAP1.

**Figure 4:** Evaluation of the effects of miR‐769‐5p/NUSAP1 axis on cell growth, apoptosis, invasion, and migration. Bladder cancer cells T24 and HT‐1376 were transfected with mimic‐NC + OE‐NC, mimic‐miR‐769‐5p + OE‐NC, mimic‐miR‐769‐5p + OE‐NUSAP1, or mimic‐NC + OE‐NUSAP1, then the following assays were carried out. A, T24 cell growth was detected by CCK‐8 assay. B, T24 cell apoptosis was detected by flow cytometry assay. C, T24 cell invasion was assessed by transwell chambers. D, HT‐1376 cell growth was detected by CCK‐8 assay. E, HT‐1376 cell apoptosis was detected by flow cytometry assay. F, HT‐1376 cell invasion was assessed by transwell chambers. G‐H, Cell migration in both T24 and HT‐1376 cell lines were detected by wound healing assay. (n = 3, ^*^ *P* < .05, compared with mimic‐NC + OE‐NC group; ^#^ *P* < .05, compared with mimic‐miR‐769‐5p + OE‐NC group)

**Figure 5:** Evaluation of the effects of miR‐769‐5p/NUSAP1 axis on cell apoptosis and EMT. A‐B, Bladder cancer cells T24 and HT‐1376 were transfected with mimic‐NC + OE‐NC, mimic‐miR‐769‐5p + OE‐NC, mimic‐miR‐769‐5p + OE‐NUSAP1, or mimic‐NC + OE‐NUSAP1, then Western blotting assay was performed to detect the protein expression levels of Bcl2, Bax, N‐cadherin, and E‐cadherin. (n = 3, ^*^ *P* < .05, compared with mimic‐NC + OE‐NC group; ^#^ *P* < .05, compared with mimic‐miR‐769‐5p + OE‐NC group)

## 4 DISCUSSION

In the current study, we reveal that miR‐769‐5p is lowly expressed in bladder cancer tissues and cells, and the low expression of miR‐769‐5p predicts shorter overall survival. In addition, we demonstrate that miR‐769‐5p exerts a tumor suppressive role in bladder cancer via binding to the 3’UTR of NUSAP1 and thereby inhibiting NUSAP1 expression.

Increasing evidences have found that miRNAs are an attractive biomarker source for cancer research as their high stability.^14^ Up to now, lots of miRNAs have been reported to be deregulated in bladder cancer and involved in cancer progression.^15^, ^16^ For instance, miR‐153 expressed at a low level in bladder cancer tissues and cells as compared with the normal tissues and cells, and low expression of miR‐153 was closely associated with advanced tumor stage and poor overall survival.^17^ They also clarified that a suppressive role of miR‐153 played in bladder cancer as miR‐153 overexpression induced cell apoptosis and repressed cell migration, invasion, and EMT and in vivo tumor xenograft growth.^17^ miR‐328‐3p was also demonstrated to be downregulated in bladder cancer, which predicted poor prognosis; miR‐328‐3p overexpression caused apparent repression in cell proliferation, migration and invasion, and EMT.^18^ miR‐146b was reported to be overexpressed in bladder cancer tissues, and silence of miR‐146b resulted in significant inhibitory effects on cell invasion and migration.^19^ The above reports indicate that miRNA can function as an oncogene or a tumor suppressive gene in the progression of bladder cancer. This study demonstrated for the first time, that miR‐769‐5p expression was downregulated in bladder cancer tissues and cell lines with the help of bioinformatics methods and RT‐PCR technology. In addition, we discovered that cell growth, migration, and invasion capacities were all repressed when miR‐769‐5p expression was increased with mimic transfection in both T24 and HT‐1376 cell lines, suggesting that miR‐769‐5p functions as a tumor suppressor in bladder cancer. By now, the roles of miR‐769‐5p in majority malignant cancers remain unclear except for non‐small cell lung cancer (NSCLC), where it exerts a tumor‐repressive role. In detail, Yang et al^20^ found that miR‐769‐5p was downregulated and associated with poor prognosis in NSCLC, and inhibited cell proliferation, migration, and invasion abilities via targeting TGFBR1 (transforming growth factor‐β1). Ma et al^21^ reported that long non‐coding RNA LINC00460 via sponging miR‐769‐5p increased the gefitinib resistance of NSCLC.

RETRACTED

Nucleolar and spindle‐associated protein 1 has been identified to play an important role in carcinogenesis. A higher expression pattern of NUSAP1 has been found in many kinds of cancers and serves as a prognostic factor, including liver cancer,^22^ breast cancer,^23^ oral squamous carcinoma,^24^ prostate cancer,^25^ pancreatic cancer,^26^ glioblastoma,^27^ and melanoma.^28^ NUSAP1 was reported to be overexpressed in bladder cancer and overexpression significantly enhanced the stemness of bladder cancer cells.^9^ To further reveal the roles of NUSAP1 in bladder cancer, we recruited the overexpressing plasmid to both bladder cancer cell lines HT‐1376 and T24. We observed that cell growth, invasion, and migration, as well as the expression of a mesenchymal cell marker, N‐cadherin were all enhanced when NUSAP1 was overexpressed, whereas cell apoptosis and the expression of an epithelial cell marker, E‐cadherin were reduced. These findings suggest that NUSAP1 functions as an oncogene in bladder cancer.

In mechanism, we confirmed that NUSAP1 was a direct target of miR‐769‐5p in bladder cancer using luciferase gene reporter assay, RT‐PCR and Western blotting technologies. Overexpression of NUSAP1 rescued miR‐769‐5p‐mediated promotions in cell apoptosis and the expression of E‐cadherin and Bax, as well as the suppressions in cell growth, migration, invasion, and N‐cadherin and Bcl2 expression, suggesting that miR‐769‐5p inhibits bladder cancer progression via targeting NUSAP1.

In conclusion, this study reveals a low expression pattern of miR‐769‐5p in bladder cancer, which closely associates with patients’ poor outcome. Furthermore, we demonstrate that via targeting the oncogene NUSAP1, miR‐769‐5p serves as a tumor suppressor in bladder cancer. These findings suggest that miR‐769‐5p/NUSAP1 axis may be a novel therapeutic target for bladder cancer.
